The article "English Word Learning Using Intelligent Massive-Scale Big Data Mining Technique" was retracted in 2023. Reasons: signs of a paper mill; suspected computer-generated content; unreliable results or conclusions; concerns about the data.

# English Word Learning Using Intelligent Massive-Scale Big Data Mining Technique

**DOI:** 10.1155/2022/6882922

**Published:** 2022-07-09

**Authors:** Lei Jin

**Affiliations:** Zhengzhou Yellow River Nursing Vocational College, Zhengzhou 450066, China

## Abstract

Big data technique has become a scientific force driving disruptive innovation and change in the education system and the entire field, including English word learning, which will undergo profound mechanism changes under the impetus of this trend. The reform of basic English education evaluation in the new era empowered by big data is an inevitable choice to get rid of the chronic problems of the “five-only” education evaluation and to implement the education that builds morality as well as learners' satisfaction. Traditional classroom teaching is combined with educational information technology to build a smart campus for English education. And data mining hidden educational information and rules are obtained to meet the requirements of students' personalized learning and other demands. However, the reality is faced with the alienation of the concept of big data in English word learning. Data mining is a very important thinking tool and learning tool, which can help students better learn basic English knowledge, memorize basic words, and improve learning effect. At the same time, it has the effect of cultivating divergent thinking and systematic learning. The foundation of English learning in high school is vocabulary. In order to help students better memorize English vocabulary, teachers can apply mind map associative memory method to implement teaching. In order to solve the problem, this paper proposes the English value concept, constructs a basic education evaluation concept empowered by big data, and eliminates teachers' concerns about technical ability. We also improve the intellectual support for evaluation reform and reasonably build a data resource platform to meet students' comprehensive quality evaluation demands. The method accurately conducts the big data evaluation to drive suggestions such as the reconstruction of educational evaluation system.

## 1. Introduction

Big data has 4V characteristics such as massive data scale (volume), diverse data style (variety), faithful data processing (velocity), and real data (veracity) [1]. More primitive basic education data information [2] strengthens and reveals a more measurable education fairness movement [3] and prefers more accurate and incomplete educational evaluation platform. It helps to smash a single evaluation type and produce more effective learners. The English word learning, as we all know, is a multiple valuation ecology, with multiple proximity and fairness issues. On October 13, the “Overall Plan for Deepening Educational Evaluation Reform in the New Era” (hereinafter referred to as the “Plan”) became the first programmatic plan to systematically solve the problem of holistic and purely guiding English education evaluation, using new data, such as pregnancy data, information technology, innovation valuation drivers, and other initiatives. In response to this principle, this work believes that it is possible to solve the problem of attaching big data to the field of English teaching evaluation, with national departments as the leading role, multiple subordinates participating the task, and instructor evaluation and judgment as the guidance of education evaluation. Data, guided by the evaluation value of the discovery data and guided by the evaluation value of the data, is the key to English learning. The normalization and inspection of evaluation activities is a guiding evaluation model and its paradigm to assist in the construction of the big data era. During the evaluation process, it is necessary to fully perform the responsibilities of nonauthoritative education evaluation and implement the evaluation effect, evaluation work, and progress and development. According to the No. 1 Municipal Regulations, we should rely on the expedient measures of school evaluation and further carry out actual civilization construction according to the evaluation content or indicators formulated by national or provincial stability. Database should be leveraged to reverse the typical problems in the rectification of authentic quasivaluation. The purpose of this exploration is to alert the demand for big data empowerment in basic education evaluation with a serious attitude, in order to handle the problems existed in the recovery of basic education evaluation big data empowerment in the era of untried. It also puts forward the research sequence and arranges the promotion of basic education evaluation. English education valuation increases and education may be beneficial.

The article "English Word Learning Using Intelligent Massive-Scale Big Data Mining Technique" was retracted in 2023. Reasons: signs of a paper mill; suspected computer-generated content; unreliable results or conclusions; concerns about the data.

In English word learning, accustomed to using the selection plane associative memory method to improve the effect of students' vocabulary learning, teachers first have to master the generation of English mind maps to promote the realization of teaching goals and to help students improving English memory. Instructors can reconcile them with actual breeding needs or order students to force word-book mind maps on their own. From the perspective of composition methods, it is mainly divided into business categories. First, according to the composition effect, the question words include pronunciation, word objects, arrangement, usage, and derivative words. This method can be utilized everywhere to capture the sincerity of the language and promote the grasp of the words. To handle this discourse, there are many English words, which can be classified and drawn; the third is to require harmony in shape. Some words in the English word book have such prefixes or affixes, which can be summarized. Fourth, according to the expressiveness of the composition, it is a pattern of synonyms or synonyms and can be generalized. ⅕ is the result of account blockchain, which saves terms in modules or textbooks and can be combined with core terms. We organize and pair English mind maps. Sixth, we have to correspond to these topics, that is, constructing related mind maps around limited topics according to the unit topics in the practice English textbooks.

English scholarship is first and chief “sign,” a purpose “classification” trial by materialize carriers such as correct, adjustments, and meanings. Acceptance of ordinary texts is important to verify the settlement of a convival kindred. A discourse is a talk emblem that charms many forms. It is the bein of cuttlefish that can describe the meaning expressed by words. Meanwhile, it can also live through the book of images. Through this text, humans can take an innocuous journey of shielded English language. In addition, it also expresses expressiveness, that is, through mental activities such as firmness, sound, and pamphlet. The symbol represents human consciousness and has meaning. For example, lively, the meaning of the two conversations is the same, but it is enough to perceive the meaning through the sound. When it occurs, our investigation evince that v] and f] are indeed homologous, more like the skirting cuttlefish. This is also like the whole of heartbeat and vent, the sounds of association. Tell the account, e.g.; f] terms are flight, mounting, fleee, flay, flay, fleet, and many others describing external enhancements, and [v] are active, very, survival, victory, love, vital, reawaken, expression, etc. The number of learners are that they allow people to identify things on the path of behavior. It is performed like onomatopoeia molt, or well-known institutions like WTO, PRC, ASAP, AD, Obama, Red Cross, CNN. Despite the anxiety of verbal memory, there are many techniques to receive English words. Whichever method is used, it is necessary to tokenize the words to obtain the vocabulary. For example, in the phonological mnemonic of rotational English memory, there is a gradual strengthening of type and meaning. With the strengthening of repetition, the English memory effect is solidified, and the word book is cultivated.

## 2. Related Work

### 2.1. Big Data Techniques

Big data has been widely used in ensuring the layout and security of smart campuses, and the unwritten campus has been transformed into a digital and perceptual campus. Through the optical analysis of pregnancy data, through the fair and appropriate means of nonwearable technologies such as face recognition, true heavy road, and intelligent early warning, the ability and level of the campus direction can be corrected. Under the same rhythm, the classroom is a field jointly created by teachers and students. The smart classroom supported by big data can break through the burden of classroom observation by teachers' physical experience and try guiding rules in the massive dynamic classroom data, making classroom teaching easier. Evaluation is more professional and intuitive, which can correct teachers' adaptability to practical tools in an interactive way and provide obligations for optimizing classroom construction and improving classroom efficiency [4]. This is not only the deep integration of information technology and classroom knowledge but also the technical cycle of teaching and breeding evaluation. Based on such classroom evaluation, teachers can more actively guide subject reflection, find education and teaching methods and the Law of Moses that are closer to students, and create a wiser classroom towards the unreal situation.

The article "English Word Learning Using Intelligent Massive-Scale Big Data Mining Technique" was retracted in 2023. Reasons: signs of a paper mill; suspected computer-generated content; unreliable results or conclusions; concerns about the data.

Although random sampling has become the capital way in the field of transformable measurement of the century, it is also a helpless choice when all data cannot be collected and analyzed and there are many reasonable flaws [5]. Traditional educational evaluation techniques have difficulty in collecting extensive and reliable data throughout the process, resulting in developmental training evaluations that are limited only in conceptual clarity. In addition, “trace data” does not truly reflect the potential of students. Only when the valuation data is detailed enough can we get close to the true state of the judges. In the bone marrow, massive data has laterally entered into new inference intervals and new problem unfolding methods [6]. Relying on big data technology, collect all-sample evaluation data to show students' hidden intelligence and laws, including comprehensively recording and scientifically promoting the cognitive and noncognitive knowledge and effect trajectory data of students' knowledge base for school opening and learning through prediction, mob, analogy mining, raw data for mortal judgment, and other methods, establish a scientific evaluation method, use the collection algorithm to mine the possible value behind the data, and solve the existing problems. Stream science can accurately diagnose, and the credibility of valuation events can be well-corrected [7]. In the topic, with the background of big data, teachers can use data mining algorithms, machine learning, regression analysis, and other learning analysis techniques to test and assemble data related to students' learning behaviors in the method of multiple measurement and multiple direct support. It can identify with oneself and students and continuously improve teaching design and teaching strategies. It changes from shaper and giver to realize the formation of knowledge with “data” and assist teaching from presupposition to reproduction. For example, back in 2007, the US pierced the “course signal engineering.” By pulling data from student prompting systems, course management systems, and serial transcripts, teachers categorize them according to their scientific performance and use data analysis techniques to identify those most likely to fail. Or stop having students adjust targeted financial services [8]. Our country can also be interested in the big league data technology. In the process of students' interactive literature, they can connect massive information sources through pipelines, use “data” to spread science, and choose borderless teaching from them. Progress visualization, in-depth mining, and analysis of multidimensional data, exploring the hidden relationship and value behind the data, implementing personalized teaching, comprehensively completing accurate services for students' energy vegetation, and improving scientific effectiveness [9].

The article "English Word Learning Using Intelligent Massive-Scale Big Data Mining Technique" was retracted in 2023. Reasons: signs of a paper mill; suspected computer-generated content; unreliable results or conclusions; concerns about the data.

### 2.2. Online Learning

Constrained by the 4V characteristics of big data, traditional data assembly and analysis techniques are unable to meet the indispensability of data expansion, forcing teachers to quickly hoard and familiarize themselves with the cognition or reasons of big data collection, analysis, cleaning, and other narratives, as well as the quality and the instruction data collection trade-off between scopes [10]. As we all know, data knowledge is a condition of data literacy disqualification. However, our rude-specific teachers exhibit data-awareness errors and crimes of insight into data. They still apply old-fashioned concepts and habits to guide their data behavioral activities. The power of data is questioned. Neither can they have a keen sense of the outstanding data and the changes in their own educational arts, nor can they fully grasp the academic structure of students for effective intervention, and cannot capture and process the narrative process and behavior of knowledge and behavior. Learn from the perspective of data and evaluation. More and more teachers are concerned about the lack of teaching and skill sickness in data warehouse. Under the distance of big data application, the old data behavior and security mechanism are gradually separated, which makes the evaluation of basic culture more accurate and scientific. However, some teachers have outdated cognitive reserves, weak scientific grouping, procedures, and weak ability to mine information from massive data, and lack of understanding of advanced data management methods and means. In particular, teachers in unsuitable fields under the setting sun are faced with the shortage of huge data and application analysis skill reserves, which directly restricts the addition and appointment of more data attention and expert richness. The survey showed that 22.7%, 38.4%, and 42.8% of Western principal and secondary teachers, respectively, were proficient in the “Scholarship Guidance System”, “Tax Student Learning Outcomes,” and “Used Spreadsheet Programs”, down from 50%. 45.0% of teachers said that they blamed it on the teaching dexterity of the corresponding information technology; 38.1% of the teachers lacked the teaching wisdom of the corresponding information technology [11]. It is important to note that most caucuses and secondary schools generally lack supporting interests and data experts to help teachers order data. Even with data blips, teachers get fewer solutions and rely more on their strengths, which does not contribute to teachers. The organizational management of teachers with diverse disciplinary backgrounds is also ambitious. Currently, unwritten data expedients present obstacles such as long collection times, inconsistent data springs, ineffective procedural data, and even poor aggregation. Analytical reasoning based on such unfinished data means can only reveal some precise or specific problems and lack comprehensiveness. Coupled with the superimposed influence of many factors such as data interruption, sluggish algorithm rules, and efficiency first, this kind of test score evaluation based on changes and restlessness limits students' character and quickly ignores students' daily performance and dynamic growth. The evolution of students needs to be “shelled” on the brand, prioritizing the broad and single development of students, and the guiding forces of educational evaluation such as educational equity, educational equity, and educational effectiveness are constantly deviating.. Traditional events become more prominent in the era of big data. In addition, the cost of expanding data construction resources is high, and the speed of big data technology update and iteration is relatively tenacious. School-failed group funds are more “struggling” to defend great data upgrades.

The article "English Word Learning Using Intelligent Massive-Scale Big Data Mining Technique" was retracted in 2023. Reasons: signs of a paper mill; suspected computer-generated content; unreliable results or conclusions; concerns about the data.

Currently, traditional data design suffers from obstacles such as time-consuming assembly, inconsistent data springs, the need for process data, or even the inability to collect them. Reanalyzing the problem on the basis of such partial data means can only show the comprehensiveness of some definite or specific trials and crimes. In addition to the superimposed advantages of many elements such as data interruption, algorithm rule black box, and efficiency priority, the friendliness of the touchstone spring evaluation with grades as the main constraint inhibits the personality of students and directly surpasses them. Maid exploitation and mobility vegetation. The education of students tend to be “unyielding-shelled” in terms of intensity, which precede to the protracted suppression of the direct power of guidebook valuation of students' range, particularity, reasonableness of manufacturing doctrine, junction of education, and effectiveness of instruction. Traditional problems are more notable in size data disposition. In addition, the excessive rib of data arrangement endowment is violent, and the success of gross data technology update and iteration is relatively indestructible. The school's inferior college funds are even more “stretched” to protect the big data upgrade.

## 3. Our Data Mining-Guided English Education

Instructors can guide students to apply the rules of association and recall of selected plants, so that they can learn English vocabulary correctly. It is necessary for students to praise the meaning, character, and technique of this recall method. On this basis, students can understand the meaning of mental map associative memory method and prominent advantages and actively use this recall law to remember violent English language [3]. The significance of this memo course is to confirm the understanding of vocabulary, promote the extraction of influential information and clues, and achieve the actual performance of retrospecting old things and learning new ones. The features of this core method are one-point memory, which supports one fixation of words, such as phonology, semantics, and spelling errors, and two-point recall, which enables the consistent relationship between two words or two types of terms to be used to reform memory. It is called the multipoint memorization, and multifaceted connections are established. Terminology can be learned on a large scale and in an orderly manner. The ingeniousness of this memory order is that one is substitution, which refers to the use of a polysemy or repetition to recover another information, such as suspicion rather than distrust. Auxiliary is monotonic, which refers to homophones related to the word book Interest memory, such as the vermin (anima) uses the homophonic memory of “shoot it to leave.” This is because this method is smoother than Chinglish. Thus, we try to use it as little as possible. The third is addition and subtraction, that is, referring to affixes or affixes and words, minus the affixes or suffixes; it becomes clear. The fourth grade is the pictographic course, which means that some descriptions are relatively brief, and you can use mental abacus to turn them into specific things, such as numbers, weeks, months, second lieutenants, and emotions. It can be found in the mind map. Moderately incorporate pictures and words to aid English word learning memory. The fifth is the immediate mode, which is more suitable for terms that are memorized directly, such as place names and other basic noun vocabulary.

The article "English Word Learning Using Intelligent Massive-Scale Big Data Mining Technique" was retracted in 2023. Reasons: signs of a paper mill; suspected computer-generated content; unreliable results or conclusions; concerns about the data.

According to the English word book that students need to memorize, teachers can let students think independently and tell the choice map of desire and utility: first obtain a mind map and then use the suggestion sketch associative recall mode to memorize more vocabulary. This objective can be given as

(1) $$\begin{array}{c} H\left(c\right)=t\left(c\right)+\underset{i}{\sum }f_{i}\left(h\right)+m. \end{array}$$

By preliminarily instructing students to use the English and delineation of associative memory rules to memorize the English word book, students can feel its significant brightness during the application process and further get used to the rules to memorize words more actively [12]. In the system to support the realization of the core of students' critical vocabulary, we give play to the value of intention planning and open thought training; instructors can also order students to adopt different teaching methods and instruct students how to expand the circle of public opinion and how to improve the memory of language. For precedents, the rules of associative memory for opinions can be divided into rough joint impression, unified joint thought, parallel association thought, classification joint consideration, causal relationship observation, and image joint thought. Different association methods have different utility. Instructors can appropriately guide students' desire for attribute associative memory method according to the specific word book. In the consolidate union fancy, use things that are close to each other to make companion associations, such as variegated synonyms or synonyms, such as a message to an office estimate, guess Malaysia via Singapore, and think via Houston Texas state. In the idea of similar association, we typically use similar things for association, such as through the east (easterly), we guess southeast (southeast), and northwest (northwest). The notion of proportion is to trigger things related to the elegance or nature of dilution according to the liking of things, especially applicable to root memo rules such as saying “nearby, around” is by-, para-, circum-, circu-, etc. Certain terminating causality can think of cause from the mainspring and cause from the effect. The Image Core approach involves combining learning content with associative concepts. As a precedent, when remembering the Great Lakes (Huron, Ontario, Michigan, Erie, and Superior), instructors can immediately extract the initials and agree to make them “home” and remain “home.” I live by the Great Lakes” method.

The article "English Word Learning Using Intelligent Massive-Scale Big Data Mining Technique" was retracted in 2023. Reasons: signs of a paper mill; suspected computer-generated content; unreliable results or conclusions; concerns about the data.

Constructing recall strategies from the data mining perspective during English word learning is a necessary condition for the formation of lexical science. This recall pattern varies from person to person, emphasizing that the use of symbols is more competitive than competition, and the recall pattern that Scholar A seems comfortable may not apply to Scholar B. There are many methods of lexical memory, including marking memory method, associative coding memory law, etymological allusions memory method called functionalist practice process, phonetic memory law, pictographic memory process, and classification resort to recall the English word teaching course in contextual memory courses. Individuals can take different approaches and symbols, which require learners to follow a method that dresses them up to learn and memorize vocabulary. Different data mining strategies are to improve language memory need to be symbolized in reading aloud. Through association, theology, and dark lessons, learners can improve their sensitivity to terms and their understanding of terms, formulas, and meanings, so as to improve and consolidate term recall, that is,

(2) $$\begin{array}{c} \text{recall}\left(i\right)=\text{mem}\left(t\right)+H\left(c\right)-f\left(j\right). \end{array}$$

First, we have to pay attention to the simplification of lexical symbols and meanings and avoid redefinition. The resymbolization of communication symbols prescribes a new interpretation and release of graphics. On the limits of strategy, we can avoid the complex and varied meanings of symbols or generate more meanings and escort texts. This will be intertwined with symbolic notices and Saturn's memory of bad words. We prove that it is necessary to update the meaning once a shabby symbol has stabilized. For example, in a bunch of words such as restrictor, sneaker, snake, and catch, it can be observed that this is a habitual firmware. Living here, you urgently need to explain the sense of English word learning, such as condensing the sn-as s-prepare snake-one action. These words are often associated with serpentine transmissions, so assigning meanings can also be more easily combined with mentioning words. Similarly, in terms of sneer, tricky, inhale, snigger, scent, snuffle, etc., this should be a feature of serpent. After union, viper and characters come to be implemented, so firmware is expanded in semiotics. Herein, if it is classified as different meanings in different memory contexts, the production and practice of memory is inhibited.

The article "English Word Learning Using Intelligent Massive-Scale Big Data Mining Technique" was retracted in 2023. Reasons: signs of a paper mill; suspected computer-generated content; unreliable results or conclusions; concerns about the data.

## 4. Experimental Results and Analysis

When comprehensively examining the many particularities of limited English learning, first use the rejection method to decompose the data to form dimensions, and Jerry has a strong common factor to return to the beginning. The sphere test is significant (chi-square utility of 5 362.943, *p* = 0.001). We can conclude that the specimen data is consistent for checking the component analysis. If the eigenvalue is greater than 1, the common factor can be at least one new variable, the variance is generally above 60%, and the common factor has too little influence on the new change. After calculation, four components with eigenvalues greater than 1 were extracted, and the variance agreement rate of these four invention variables was 63.672%. Again, the kinds and factors of element rotation that must be taken out at this rate, such as making source substitutions, have the largest charge value on a particular agent and most similar charge values on other factors and local characteristics that improve fecal sticks to ordinary hoagie to facilitate inferior elements. The component loads and common grades obtained by the highest dispute rotation method in this consideration are shown in Table 1. Among them, factor 1 contains 9 new allusions, and the item level involves dialect wisdom, language spirit, and literary skill. Therefore, the famous ontology learning endures three factors that limit the 3 original sub-2s that mainly involve extracurriculars.

Finally, the composition coefficient matrix is calculated by the regression method, and the goodness of each sample on the factor is obtained. Since each element is the calm of the noble agent load, each prospect is obtained by four factors. The agent with the most load can be considered as the most serious language clothing of the sample, which can be of interest as the main feature of the sample, and thus the subdivision dictionary. After statistics, a total of 147 people scored the highest. The proportion of students who mainly focus on stylistic needs, entertainment needs, and degree examinations is relatively high, and there is no imbalance. However, it is also the maximum luminosity of the sample. Different combinations must be different. For example, the limit of the attempt is -1, while the limit of another sample is 1. Only the latter can really show that the game has a muscular performance in the game. Therefore, it is superior when the value of the common element is greater than 1; the trypiece has the following language: learning needs, beyond the commonality; the results are shown in Table 1. It can be seen that the students' mediety is high in all four element dimensions, with 31 students. There are obvious features in one degree, and another 9.52% of students have obvious shapes in two proportions.

The article "English Word Learning Using Intelligent Massive-Scale Big Data Mining Technique" was retracted in 2023. Reasons: signs of a paper mill; suspected computer-generated content; unreliable results or conclusions; concerns about the data.

Since only one pure substitution is studied when calculating the maximum substitution score, and factors greater than 1 are the scarcity of the other three factors, the ubiquitous speech habit problem situation needs to be decomposed. Furthermore, the method deals with the specific characteristics of the sample. So segmentation habit is hopeless; it is just one aspect of data mining in education and letters (17 : 35%). However, elemental analysis converts high-dimensional data with 13 variables into dimensional data; it can hurry up aggregate class analysis (17e 252%). In view of this, this observation fabricates a K-means group plan and uses the four-agent motivation of the samples as a variable to crowd the samples. The object is to further subdivide the patterns that are in harmony with the character characteristic of each sample. Linguistics must be lobate into several categories. This order is the most clustering method based on numerical variables. The number of groups that need the Benton's experience is based on the number of joint common factors, the number of mobs from 3 to 3, and the 5 categories firmly. The factors of each group were obtained and marked. In the same way, the rise of thugs is expressed with the items of meridian factor reasons (distinguished in black italics). It can be found that when the crowd results in five classes, gate 1 and division 2 are the largest among factor 3 and class 3, and classes 3 and 4 have the highest motivation on agent 4, while group 5 has the highest motivation on agent 4. 4 has the highest score on factor 1; when the aggregation is terminated to four categories, there are still two categories with the highest score on factor 4; other high-scoring categories fall on component 3 and substitute 1. This is difficult for five-category crowd events. When the clustering results in three classes, the high subordination statement is a reflection of factor one, factor three, and factor four. It can be seen that the clustering results of the four types and five emblems are correct, and the clustering results of the three types have been further purified. Therefore, it is more appropriate to classify all patterns into three categories. It can be measured that the strength of the first category of English learning will inevitably be reflected in the future, while the majority of the need for dilemma 2 is classroom inspection, and the main requirement of the third category of the group is the acquisition of vocabulary. No matter which category it is, agent 2 is very demanding., Mingyu's request came last in the interviews of vocational students.

The article "English Word Learning Using Intelligent Massive-Scale Big Data Mining Technique" was retracted in 2023. Reasons: signs of a paper mill; suspected computer-generated content; unreliable results or conclusions; concerns about the data.

## 5. Conclusions

The meaning of semiotics for vocabulary acquisition and memory and the basic basis of experiential learning of symbols for learning are described in the following, or in other words, it integrates symbolic thinking, thus completing the conversion between language meanings. From the above analysis, we should see that the multidimensional conversion and interpretation of symbols to words has also created the complexity of symbols themselves, so there is the problem of the maximum benefit of symbol coding, that is, although the vocabulary learning and memory of semiotics has theory. However, it also has its own applicable limits in terms of human spiritual cognition. In a word, no matter what method of vocabulary acquisition and memory is used, in terms of symbols themselves, the task of vocabulary acquisition can only be truly accomplished and semiotics be put into practice only when there is an easily accepted proof of the connection between vocabulary and meaning.

## Figures and Tables

**Table 1:** Important associative rules.

Consequent	Antecedent	ID	Instance	Learning rate
Female	4.5	61	73	51.212%
Male	3.7	16	21	32.443%
Male	2.6	13	44	27.678%
Female	6.5	32	65	25.448%
Male	3.4	9	71	32.879%
Female	1.7	10	17	19.485%
Female	4.5	32	54	27.470%

## Data Availability

The data used to support the findings of this study are available from the corresponding author upon request.
